This article has been retracted.

# Comparison of Two Surgical Approaches to Supination-External Rotation-Type Ankle Fractures

**DOI:** 10.1155/2022/7726726

**Published:** 2022-04-11

**Authors:** Bingqian Chen, Zhengfei Wang, Zhi Chen, Xiaohong Qu, Xiaowen Fang, Xuesong Wang, Guoxiu Ke

**Affiliations:** Department of Orthopaedics, Changshu Hospital Affiliated to Soochow University, First Peoples' Hospital of Changshu City, Changshu 215500, Jiangsu, China

## Abstract

**Objective:**

To compare the clinical outcome and postoperative complications of the treatment of supination-external rotation-type ankle fractures using the posterolateral approach in the prone position and the lateral approach in the supine position.

**Methods:**

A retrospective cohort study was conducted in our hospital, including a total of 66 patients ranging from January 2013 to February 2016, regardless of age or sex. All the patients were classified as Lauge-Hansen supination-external rotation (SER)-type ankle fractures and were assigned to receive an open reduction and internal fixation (ORIF) through a posterolateral approach performed in the prone position (the “posterolateral approach group,” 32 patients), or a lateral approach performed in the supine position (the “Lateral Approach Group,” 34 patients). In the posterolateral approach group, 5 patients had Grade II fractures, 8 had Grade III fractures, and 19 had Grade IV fractures; among whom, 12 underwent fixation of the posterior malleolus with hollow screws and 6 with plates, and none of them had fixation of the distal tibiofibular syndesmosis; in the lateral approach group, 4 patients had Grade II fractures, 12 had Grade III fractures, and 18 had Grade IV fractures; among whom, 21 received fixation of the posterior malleolus, and 5 received fixation of the distal tibiofibular syndesmosis. The postoperative complications and ankle scores were recorded.

**Results:**

After 1 year of follow-up, in the posterolateral approach group, the incision healed by primary intention and sutures were removed 2 weeks after the operation in all patients; 1 patient had pain in the region posterior to the fibula, presumably peroneal tendon irritation induced by internal fixation, which disappeared after fracture union and fixation device removal; no loosening or breakage of the internal fixation device was reported; the rate of good to excellent results was 96.8% at 12 months. In the lateral approach group: 1 case of wound infection, 1 case of necrosis of lateral skin flap, and 3 cases of lateral skin irritation were reported; the rate of good to excellent results was 94.6% at 12 months.

**Conclusion:**

Compared with the traditional lateral approach, the posterolateral approach for the reduction and internal fixation of supination-external rotation-type ankle fractures performed in the prone position has more satisfactory clinical outcomes, with better reduction, more secure fixation, and smaller wound.

## 1. Introduction

In supination-external rotation-type ankle fractures, which may be complicated by posterior and medial malleolus fractures, the fibular fracture line is at the level of the distal tibiofibular syndesmosis, running from anteroinferior to posterosuperior, and the distal fractured bones have a tendency of posterior lateral dislocation [1, 2]. Traditionally, it is treated by reduction and placement of a plate lateral to the fibula through the lateral approach; the concurrent posterior malleolus fractures are usually reduced indirectly and fixed with hollow screws turned anterior to posterior. This approach has significant disadvantages [3]. First, the plate placed laterally to the fibula cannot prevent the tendency of posterolateral dislocation of the distal fractured bones. Also, the approach and position used will not allow direct reduction and effective fixation of posterior malleolus fracture, weakening reduction effect, and fixation strength. To overcome the aforementioned disadvantages, the posterolateral approach to the ankle is introduced in the treatment of supination-external rotation-type ankle fractures. This approach allows the placement of the plate posterior to the fibula, providing better support. It also allows directly the revealing of the posterior malleolus fractures for secure fixation [4]. We compared the clinical outcome of the treatments using the new posterolateral approach in the prone position and the conventional lateral approach in the supine position performed in our hospital from January 2013 to February 2016 and reported as follows.

The purpose of this study mainly contains 3 aspects. First, from this study, we were able to determine whether the posterior lateral approach in the prone position is more convenient than the traditional lateral approach. Second is which of the two surgical approaches has smaller incision and less trauma. Thirdly, whether the prone posterior lateral approach is more effective and has fewer postoperative complications compared to the traditional lateral approach. These three points are the most important concerns of surgeons. Through this study, it can be concluded that surgical procedure is more suitable for the treatment of supination and external rotation fracture and is more worthy of clinical promotion. At the same time, we hope to find the advantages and disadvantages of this new technology and find the details that need to be paid attention to during the operation. This is conducive to the application and promotion of the new technology and the improvement of the treatment level of ankle fractures.

## 2. Materials and Methods

### 2.1. General Information

A total of 66 patients with Lauge-Hansen supination-external rotation (SER)-type ankle fractures were included in this study. The inclusion criteria include ① aging from 25 years old to 70 years old; ② no serious medical diseases, such as hypertension and diabetes, can tolerate surgery; ③ complete medical records and follow-up data were available. The exclusion criteria include ① age under 25 years old and over 70 years old; ② patients with severe medical conditions who are unable to tolerate surgery; ③ lack of complete medical records and missing visitors. Of which 32 patients, 18 males and 14 females, aged 34–66 years (mean age 43 years), were assigned to the posterolateral approach group, of whom, 5 were classified as Grade II fractures, 8 were Grade III fractures, and 19 were Grade IV fractures. The remaining 34 patients, 16 males, and 13 females, aged 27–61 years (mean age 42 years), were assigned to the lateral approach group, of whom 4 were Grade II fractures, 12 were Grade III fractures, and 18 were Grade IV fractures.

The patients were given symptomatic treatment, such as elevation of the fractured ankle and application of an ice pack. Routine anteroposterior and lateral radiographs and CT scanning of the ankle were performed prior to the surgery, to determine the morphology and dislocation of the fractured ankle. The surgeries were performed 5–10 days after the injury when the swelling had significantly improved, and local dermatoglyphic appeared.

### 2.2. Operation Methods

Spinal anesthesia or epidural anesthesia is administered, and a tourniquet is applied at the root of the thigh. For patients in the posterolateral approach group, the patient was placed in the prone position, with cushions placed under the hip and knees. After routine disinfection and draping, a longitudinal incision was made at the midline between the posterior border of the fibula and the lateral border of Achilles's tendon, extended beyond the tip of the lateral malleolus distally. The skin was carefully cut open to protect the sural nerve and small saphenous vein in the subcutaneous fascia. Then, the deep fascia was incised, and the insertion of flexor hallucis longus on the fibula was dissected sharply and pulled medially to reveal the posterior malleolus and distal posterior tibiofibular ligament. A blunt dissection was made lateral to the tendon of peroneus longus and peroneus brevis, and the muscle was pulled medially to reveal the underlying fibula, which was done carefully to protect the peroneal retinacula located on the distal aspect of the fibula. The posterior malleolus fracture was reduced first and fixed with hollow screws or a support plate (with hollow screws in 21 patients and with plate in 6 patients); then, the fibula was reduced and fixed with a highly plastic reconstruction plate placed posteriorly to the fibula. For patients with concurrent medial malleolus fractures, an arc-shaped incision was made in the medial aspect of the ankle to reveal the medial malleolus fracture, which was reduced and fixed with hollow screws (Figures 1 and 2).

For patients in the lateral approach group, the patient was placed in the supine position, with a sandbag placed under the hip on the affected side. After routine disinfection and draping, a longitudinal incision was made laterally to the fibula, and advanced layer by layer, to reveal the fibula fracture. After removing the soft tissues in the fractured bone, the manual reduction was performed followed by temporary fixation with Kirschner wires, and then, a highly plastic reconstruction plate was placed laterally to the fibula and fixed with screws. For patients with concurrent medial malleolus fractures, an arc-shaped medial incision was made to reveal the medial malleolus fracture, and then, the anatomical reduction was performed followed by fixation with 1–2 hollow screws. For posterior malleolus fractures involving >1/4 of the joint (20 patients), fixation with 1–2 hollow screws placed from posterior to anterior was performed (Figure 3).

A hook test was performed for patients from both groups. For patients identified with the instability of the distal tibiofibular syndesmosis (5 in the lateral approach group and 0 in the posterolateral approach group), the distal tibiofibular syndesmosis was reduced using reduction forceps and fixed with 1–2 cortical bone screws placed from the fibula during ankle dorsiflexion.

After the surgery, patients were given the elevation of the fractured ankle and the application of an ice pack for 48 hours. They started functional training after the removal of vacuum drains the next day and had sutures removed at 2 weeks when their wounds healed. At 2 months, the screws for fixation of distal tibiofibular syndesmosis were removed. Radiographs were obtained, and ankle function scores (American Orthopedic Foot and Ankle Society, AOFAS) and complications were recorded during the follow-up visits at 3, 6, and 12 months.

AOFAS: in 1994, the American Association of Foot and Ankle Society (AOFAS) developed and recommended the AOFAS Ankle-Hindfoot Scale, including the fill and physician examination, a total of nine projects: indicators have pain, function and autonomic activities, support conditions, the biggest walking distance, ground to walk, before and after the abnormal gait, activity (flexing and stretching), hind activities (varus and valgus), ankle—after sufficient stability (and varus and valgus) before and after, the foot line of force. Grading standard: >90, excellent; 75–89, good; 50–74, fair; <50, poor.

### 2.3. Statistical Analysis

Statistical analysis was performed using SPSS 21.0 (Statistical Package for Social Sciences. SPSS Inc. Released 2010, SPSS Statistics for Windows, Version 21.0, Chicago: SPSS Inc.). Measurement data were present as *x*^−^ ± *s*. The mean AOFAS scores and standard deviations of each group were calculated and compared with each other using the Mann–Whitney *U* test. Logistic regression was used to see if a combination of factors including sex, fracture type, and classification of the fracture might have influenced the AOFAS scores for each group. Statistical significance was defined as *P* < 0.05.

## 3. Results

All patients were followed up for at least one year, both in the clinic and by telephone. Follow-up mainly included wound healing, postoperative pain, and ankle function recovery. In the posterolateral approach group, the incision healed by primary intention and sutures were removed 2 weeks after the operation in all patients. In the lateral approach group, 1 patient had a wound infection at 1 week and was treated with debridement with continuous closed irrigation, and the sutures were removed 2 weeks later when the wound healed; 1 patient developed necrosis of lateral skin flaps, and with increased frequency of dressing changes, the wound healed under scabbing.

All patients were followed up for 12 months, during which, 1 patient from the posterolateral approach group felt mild pain in the region posterior to the fibula, possibly due to irritation of the peroneal tendon by the fixation plate, which disappeared after fracture union and fixation device removal; 3 patients reported pain and discomfort in the lateral skin due to irritation by the plates, which disappeared after the removal of the plates; no loosening or breakage of the internal fixation device or redisplacement of fractures was reported.

The ankle function scoring (AOFAS) at 12 months showed 23 excellent results, 8 good results, and 1 poor result, with a rate of good to excellent results of 96.8%, in the posterolateral approach group; and The ankle function scoring (AOFAS) at 12 months showed 22 excellent results, 10 good results, and 2 poor results, with a rate of good to excellent results of 94.1%, in the lateral approach group (Tables 1 and 2).

## 4. Discussion

### 4.1. Characteristics of Supination-External Rotation-Type Ankle Fractures

Supination-external rotation-type ankle fractures are commonly seen in clinical practice, accounting for about 85% of all ankle fractures [5]. It has the following characteristics [1, 2]: first, the broken end of the fibula is located in the distal tibiofibular syndesmosis, the fracture line running obliquely from anteroinferior to posterosuperior; second, the distal fractured bones have the tendency of posterior lateral dislocation.

Supination-external rotation-type ankle fractures are usually complicated by posterior malleolus fractures. The posterior malleolus is an important part of the articular facet on the tibia, whose displacement may lead to a decreased area of the articular surface, and concentration of joint stress [6, 7]. Also, it gives attachment to the distal posterior tibiofibular ligament. Therefore, the normal attachment of the distal posterior tibiofibular ligament relies on a normal anatomical position of the posterior malleolus, and maintaining the distal posterior tibiofibular ligament tension is essential for the stability of distal tibiofibular syndesmosis, especially when the medial ankle is injured [8, 9]. In conclusion, the posterior malleolus is important for the integrity and stability of the ankle [10–12]. In this study, hollow screw or reconstruction plate fixation following routine revealing and reduction of posterior malleolus fracture was performed for patients in the posterolateral approach group, and indirect reduction and fixation of posterior malleolus fracture were performed for 21 patients from the lateral approach group, and no case of instable distal tibiofibular syndesmosis was reported.

Posterior malleolus fracture can be fixed with hollow screws or support plates in the treatment through a posterolateral approach. In this study, 21 patients had screw fixation, and 6 had plate fixation, both achieved a satisfactory effect, with no case of redislocation reported, and showed no significant difference in 1-year satisfaction with clinical outcomes. However, the screw fixation is better compared to the plate fixation, as it permits smaller wound, simpler operation, and lower cost. Therefore, we recommend the screw fixation for posterior malleolus fracture.

### 4.2. Two Treatment Options and Their Advantages and Disadvantages

The lateral approach in the supine position, which allows the surgeon to reach the fracture site from a lateral incision, and placement of plates lateral to the fibula, is currently widely used in the surgical treatment of ankle fractures, as it is easy to learn and convenient for the management of medial malleolus fractures [13]. However, it has many disadvantages. First, through this approach, the posterior malleolus is not revealed and can only be reduced indirectly and fixed with hollow screws turned anterior to posterior, producing poor reduction and fixation. Second, this approach does not allow the placement of a plate posterior to the fibula, which provides better support. Finally, the plate placed underneath the skin lateral to the fibula may cause irritation of the skin, or even necrosis of flaps. In this study, 3 patients from the lateral approach group experienced skin irritation from the plates, which was relieved after the removal of the plates.

The posterolateral approach in the prone position allows the revealing of the lateral and posterior malleolus through an incision, facilitating better management of supination-external rotation-type ankle fractures [14, 15]. First of all, it allows the placement of a lateral plate posterior to the fibula, which provides better support and is more conformable to the principle of biomechanics [4]. Second, posterior malleolus fracture is revealed from the same incision, allowing better reduction and more secure plate or screw fixation. Also, the placement of a plate deep in the soft tissues helps to avoid skin irritation and reduce the risk of flap necrosis. As evidence, in this study, no patient from the posterolateral approach group experienced flap necrosis, while 1 case of flap necrosis and 1 case of wound infection were reported in the lateral approach group. In addition, with the posterior plate placement and anterior-to-posterior screw fixation, there is no concern about screws in the articular cavity, allowing for bicortical fixation with long screws, which has a higher resistance to pull-out and is particularly suitable for osteoporotic elderly patients [16]. Finally, the prone position is helpful for the reduction of fractures. We noticed a phenomenon in clinic practice that the fracture block of lateral malleolus, even if comminuted, has had a good reduction when revealed through the posterolateral approach,which is possibly due to the action of gravity, which places the ankle in dorsiflexion and a neutral position, and corrects external rotation and dislocation.

The results of this study showed that, although the posterolateral approach was more beneficial for the reduction and fixation of fractures, and the posterolateral approach group reported fewer cases of complications than the lateral approach group, there was no significant difference in the 1-year satisfaction with clinical outcomes between the two groups.

### 4.3. Considerations for Surgeries through Posterolateral Approach

First, the sural nerve shall be carefully protected during the operation. The sural nerve lies on the posterolateral side of the ankle under the skin, usually crossing the lower segment of the incisions from posterior to anterior, and thus shall be protected when dissecting the fat layer [17, 18]. Second, note that the insertion of flexor hallucis longus on the fibula should be dissected and pulled medially, to reveal the posterior malleolus fractures, during which the posterior tibial vessels and nerves immediately medial to it shall be protected [19]. Third, when revealing the posterior malleolus fracture, be careful not to cut the distal tibiofibular ligament attached to it. In addition, the plates shall not be placed too low but placed above the groove for the peroneal tendon, or irritation of the tendon will occur [20]. In this study, a patient from the posterolateral approach group experienced pain in the region posterior to the fibula, which is possibly caused by irritation of the peroneal tendon by the fixation plate placed too low. What's more, a thin plate with good plasticity shall be chosen to reduce the risk of tendon irritation. Usually, a 3.5 mm reconstruction plate or 1/3tubular plate is preferred. Finally, a hook test before the end of the surgery is necessary for determining whether the distal tibiofibular syndesmosis is stable enough. If the distal tibiofibular syndesmosis is unstable despite the fixation of posterior malleolus, which is more common in cases complicated by medial collateral ligament rupture, screw fixation of the distal tibiofibular syndesmosis is required. In this study, 5 patients from the lateral approach group, who did not receive the fixation of posterior malleolus due to small sizes, were identified with unstable distal tibiofibular syndesmosis in the hook test, which was corrected by screw fixation of the distal tibiofibular syndesmosis.

## 5. Conclusion

Compared with the traditional lateral approach, the posterolateral approach in the prone position allows the revealing of the lateral and posterior malleolus through an incision and better reduction and fixation of the posterior malleolus. It also allows the placement of the lateral plate posterior to the fibula, which provides better mechanical support and helps to avoid skin irritation. This is a safe and excellent surgical technique to treat supination-external rotation-type ankle fractures and has more satisfactory clinical outcomes, with better reduction, more secure fixation, and safer wound than the traditional lateral approach, though there is no significant difference in 1-year satisfaction rate. In the posterolateral approach group, there was no significant difference in clinical efficacy and complication rates between the lag screw and the plate fixation for posterior malleolus. However, the use of hollow screws permits smaller wound, simpler operation, and lower cost.

In future work, we will strive to constantly improve the technology of the posterolateral approach in prone position to treat supination-external rotation-type ankle fractures. At the same time, we will also apply this technology to other types of ankle fractures, compare it with the traditional surgical methods, and analyze the advantages and disadvantages of the technology.

## Figures and Tables

**Figure 1:** (a–h) The procedure of posterolateral approach for pronation-extorsion fractures of the ankle. (a) Patients took a prone position. (b) The sural nerve lies on the posterolateral side of the ankle under the skin, usually crossing the lower segment of the incisions from posterior to anterior. (c) Pulled flexor hallucis longus medially to reveal the posterior malleolus. (d) The tendon of peroneus longus and peroneus brevis was pulled medially to reveal the underlying fibula. (e) The fibula was reduced and fixed with a highly plastic reconstruction plate placed posteriorly to the fibula. (f, g) The posterior malleolus fracture was reduced and fixed with a support plate or a hollow screw. (h) An arc-shaped incision was made in the medial aspect of the ankle to reveal the medial malleolus fracture, which was reduced and fixed with hollow screws.

**Figure 2:** (a, b) 45-year-old female patients with right ankle fracture caused by trauma. (c–h) CT scan shows that the fracture involves medial, lateral, and posterior malleolus. The fracture belongs to the supination-external rotation-type (Grade IV). (c–f) The prone position and posterolateral approach were used. The fibula was fixed by a plate, the posterior malleolus was fixed by a lag screw, and the medial malleolus was fixed by two hollow screws. (h, i) One year after surgery, the X radiographs show that the fractures were healed well and the ankle function recovered excellently.

**Figure 3:** (a, b) A 47-year-old male patients with a right ankle fracture caused by trauma. (c, d) CT scan shows that the fracture involves medial-lateral and lateral malleolus. The fracture belongs to the supination-external rotation-type (GradeIII). (e, f) The supine position and lateral approach were used, a plate was used to fix the lateral malleolus, and two lag screws were used to fix the medial malleolus. (g, h) One year after surgery, the X radiographs show that the fractures were healed well, and the ankle function recovered excellently.

**Table 1:** Personal information and rates of excellent results in both groups.

Group	*n*	Mean age	Presence of concurrent posterior malleolus fracture	Use of screws at the distal tibiofibular syndesmosis	Rates of excellent results (%)
Posterolateral approach group	32	43	27	0	96.8
Lateral approach group	34	42	30	5	94.1

**Table 2:** Rates of excellent results of different treatments of posterior malleolus fractures through a posterolateral approach.

Group	*N*	Mean age	Male	Female	Rates of excellent results (%)
Hollow crew fixation	21	46	7	5	95.4
Plate fixation	6	43	3	4	94.6

## Data Availability

The dataset used to support the findings of this study is available from the corresponding author upon request.
